This article has been retracted.

# Natural product pectolinarigenin inhibits osteosarcoma growth and metastasis via SHP-1-mediated STAT3 signaling inhibition

**DOI:** 10.1038/cddis.2016.305

**Published:** 2016-10-13

**Authors:** Tao Zhang, Suoyuan Li, Jingjie Li, Fei Yin, Yingqi Hua, Zhouying Wang, Binhui Lin, Hongsheng Wang, Dongqing Zou, Zifei Zhou, Jing Xu, Chengqing Yi, Zhengdong Cai

**Affiliations:** 1 Department of Orthopaedics, Shanghai General Hospital, Shanghai Jiao Tong University School of Medicine, Shanghai, China; 2 The Institute of Cell Metabolism and Disease, Shanghai Key Laboratory of Pancreatic Cancer, Shanghai General Hospital, Shanghai Jiao Tong University School of Medicine, Shanghai, China

## Abstract

Signal transducer and activator of transcription 3 (STAT3) has important roles in cancer aggressiveness and has been confirmed as an attractive target for cancer therapy. In this study, we used a dual-luciferase assay to identify that pectolinarigenin inhibited STAT3 activity. Further studies showed pectolinarigenin inhibited constitutive and interleukin-6-induced STAT3 signaling, diminished the accumulation of STAT3 in the nucleus and blocked STAT3 DNA-binding activity in osteosarcoma cells. Mechanism investigations indicated that pectolinarigenin disturbed the STAT3/DNA methyltransferase 1/HDAC1 histone deacetylase 1 complex formation in the promoter region of SHP-1, which reversely mediates STAT3 signaling, leading to the upregulation of SHP-1 expression in osteosarcoma. We also found pectolinarigenin significantly suppressed osteosarcoma cell proliferation, induced apoptosis and reduced the level of STAT3 downstream proteins cyclin D1, Survivin, B-cell lymphoma 2 (Bcl-2), B-cell lymphoma extra-large (Bcl-xl) and myeloid cell leukemia 1 (Mcl-1). In addition, pectolinarigenin inhibited migration, invasion and reserved epithelial–mesenchymal transition (EMT) phenotype in osteosarcoma cells. In spontaneous and patient-derived xenograft models of osteosarcoma, we identified administration (intraperitoneal) of pectolinarigenin (20 mg/kg/2 days and 50 mg/kg/2 days) blocked STAT3 activation and impaired tumor growth and metastasis with superior pharmacodynamic properties. Taken together, our findings demonstrate that pectolinarigenin may be a candidate for osteosarcoma intervention linked to its STAT3 signaling inhibitory activity.

Osteosarcoma is the most common malignant bone tumor in children and adolescents and arises from cells of mesenchymal osteoblast origin.^1, 2^ Despite advances in surgery and multiagent chemotherapy, nearly 30% of patients still die from osteosarcoma.^2^ And the survival rates for osteosarcoma remain relatively low over the past two decades.^3^ Therefore, it is necessary to develop novel therapeutic approaches for osteosarcoma treatment.

Signal transducer and activator of transcription 3 (STAT3) is an important transcription factor that involves in proliferation, survival, apoptosis, angiogenesis and metastasis.^4, 5^ Upon stimulation by cytokines (interleukin-6 (IL-6), IL-11 and etc.) and growth factors (EGF, PDGF and etc.), STAT3 can be phosphorylated at tyrosine residue 705. STAT3 phosphorylation facilitates its homo- and heterodimerization, and the dimer then enters the nucleus where it regulates transcription, leading to increased downstream gene transcription such as *Vegf*, *Bcl-2*, *BcL-xL*, *Survivin, XIAP*, *MMPs* and etc.^6^ Src homology region 2 (SH2) domain-containing phosphatase 1 (SHP-1) belongs to a family of non-receptor protein tyrosine phosphatases (PTP) and acts as a negative regulator of numerous signaling pathway.^7^ Previous studies reported SHP-1 tyrosine phosphatase inhibited JAK/STAT3 signaling and contributed to antitumor activity in a wide variety of tumor.^8, 9^ Recent studies have indicated that STAT3 is constitutively activated in many cancers, including, but not limited to, head and neck squamous cell carcinoma (HNSCC),^10^ breast cancer,^11^ ovarian cancer,^12^ lung cancer^13^ and leukemia.^14^ With respect to osteosarcoma, the expression level of p-STAT3 is strongly associated with its prognosis and approximately 20% osteosarcoma was shown to express high levels of p-STAT3^Tyr705^.^15^ The activated STAT3 pathway is vital for cell growth and metastasis of human sarcoma.^16^ Consequently, STAT3 pathway may represent a target for therapeutic intervention in osteosarcoma.

A variety of inhibitors of STAT3 have shown to inhibit tumor cell growth and metastasis both *in vitro* and *in vivo*.^17, 18^ Agents derived from natural sources have gained considerable attention from researchers and clinicians because of their safety, efficacy and immediate availability, and they are the best sources of drugs and drug leads for novel drug discovery. Natural agents, such as Cucurbitacin E,^19^ Galiellalactone,^20^ Atiprimod^21^ and betulinic acid,^9^ have shown significant efficacy in blocking STAT3 activation. Pectolinarigenin, a flavonoids compound, which can be isolated from the aerial parts of *C. chanroenicum* has been shown to possess numerous biologic activities such as anti-inflammation and anti-allergy.^22, 23^ Some research also reported pectolinarigenin repressed cancer growth *in vitro*, including lung cancer, hepatocellular carcinoma, melanoma and colorectal adenocarcinoma.^23^ However, the function and regulatory mechanism of pectolinarigenin in osteosarcoma growth and metastasis are still not well understood.

In our current study, we used a dual-luciferase assay to reveal the natural product pectolinarigenin counteracted STAT3 activity. We found pectolinarigenin inhibited constitutive and IL-6-induced STAT3 phosphorylation and blocked STAT3 DNA-binding activity and blocked STAT3 cyoplasmic-to-nuclear translocation in osteosarcoma cells. We also showed pectolinarigenin blocked a transcription repression program composed of STAT3/DNA methyltransferase 1 (DNMT1)/HDAC1 histone deacetylase 1 (HDAC1), thus restoring the expression of STAT3-negative mediator SHP-1. Functional assays and western blot analyses indicated pectolinarigenin suppressed osteosarcoma cell growth, motility and reduced the expression of STAT3 related proteins. We further demonstrated the inhibitory efficacy of pectolinarigenin in osteosaocma growth and metastasis using preclinical animal models. In conclusion, these findings implied pectolinarigenin can act as an anticancer agent in osteosaocma via inhibiting STAT3 signaling.

## Results

### Pectolinarigenin inhibits STAT3 signaling in osteosarcoma

STAT3 is constitutively activated and prognostic value has been identified to associate with the phosphorylated STAT3-signatures in osteosarcoma. As such, targeting STAT3 signaling with small molecule inhibitors is an emerging therapeutic strategy for osteosarcoma. Screening with a dual-luciferase reporter assay, we identified a flavonoids compound, pectolinarigenin (MW: 314.29), with STAT3 inhibitory activity in a dose-dependent manner in our internal Chinese medicine chemical library (Figure 1a). The chemical structure of pectolinarigenin was shown in Figure 1b. Immunoblotting with an antibody recognizing p-Tyr705 residue of STAT3 showed the constitutive activation of STAT3 was blocked by pectolinarigenin (Figure 1c). In response to growth factor or cytokine stimulation, p-Tyr705 residue of STAT3 can also be activated. IL-6 represents one of the most important inflammatory factors inducing STAT3 phosphrylation at Tyr705.^24^ Our results indicated pectolinarigenin significantly suppressed IL-6-induced STAT3 phosphrylation (Figure 1d). Intriguingly, Janus kinase 2 (JAK2), the known upstream regulatory signal of STAT3, was inactivated by pectolinarigenin (Figures 1c and d). Constitutive or inducible activation of STAT3 Tyr705 is critical for its biologic function, as it facilitates STAT3 dimerization, further promoting STAT3 cytoplasimic-to-nuclear translocation.^25^ We found IL-6-induced STAT3 nuclear accumulation was largely impaired after pectolinarigenin treatment (Figure 1e). Similar results were observed when immunobloting with an anti-STAT3 antibody to detect STAT3 distribution in both cytoplasm and nucleus (Figure 1f). In addition, the results of an electrophoretic mobility shift assay (EMSA) confirmed that treatment with pectolinarigenin led to a dose-dependent inhibition of STAT3 DNA-binding activity in 143B cells (Figure 1g). These results showed pectolinarigenin is a potent inhibitor of STAT3 signaling in osteosarcoma.

### SHP-1 is essential for pectolinarigenin-mediated STAT3 Tyr705 phosphrylation repression

PTPs have been implicated in STAT3 signaling activation,^26^ and we sought to investigate whether PTPs involved in the blockade of STAT3 signaling by pectolinarigenin in osteosarcoma cells. Sodium vanadate, a nonspecific phosphatase inhibitor, could reverse pectolinarigenin-induced inhibition of STAT3 activity (Figure 2a), implying the involvement of tyrosine phosphatases. We thus detected the protein level of several protein phosphatases (SHP-1, SHP-2 and phosphatase and tensin homolog (PTEN)) after pectolinarigenin exposure. We found pectolinarigenin specifically increased SHP-1 expression, whereas it had no effect on the expression of SHP-2 and PTEN (Figure 2b). This result suggested SHP-1 has an important role in pectolinarigenin-induced inhibition of STAT3 activity. Next, we queried whether pectolinarigenin treatment could induce SHP-1 at the transcriptional level. As anticipated, SHP-1 mRNA was significantly increased when treated with pectolinarigenin (Figure 2c). These data suggested that the upregulated SHP-1 protein expression may be caused by an increase at transcriptional level. Previous studies reported STAT3 nucleates a transcriptional repressive complex composed of DNMT1 and HDAC1 in SHP-1 promoter site, thus leading to the silencing of SHP-1 in cancers.^27^ Therefore, we explored the effect of pectolinarigenin on STAT3/DNMT1/HDAC1 complex formation in 143B nuclear lysates. As shown in Figure 2d, after immunoprecipitating STAT3, we detected the reduced associated DNMT1 and HDAC1 when treated with pectolinarigenin. Similarly, after immunoprecipitating DNMT1, the associated STAT3 and HDAC1 decreased. Quantitative ChIP (qChIP) analysis in 143B cells using specific antibodies against STAT3 and DNMT1 showed a release of STAT3 and DNMT1 on the SHP-1 promoter after pectolinarigenin treatment (Figure 2e). These data demonstrated that pectolinarigenin induced SHP-1 expression by reducing the STAT3/DNMT1/HDAC1 complex on SHP-1 promoter in osteosarcoma. To validate the important effect of SHP-1 on pectolinarigenin-induced inhibition of STAT3 activity, we silenced SHP-1 with small interfering RNA (siRNA) duplex in 143B cells (Supplementary Figure 1). We used siRNA-1 to perform the following experiment as the knockdown efficiency remained the same in two pairs of siRNAs. As expected, downregulation of SHP-1 by siRNA-1 abolished the inhibitory effects of pectolinarigenin on STAT3 p-Tyr705 (Figure 2f, up panel). The viability of tumor cells was also partly increased by ablation of SHP-1 (Figure 2f, low panel). In addition, ectopic expression of SHP-1 in 143B cells downregulated STAT3 p-Tyr705 level and decreased cell viability (Figure 2g). These data indicated SHP-1 has a critical role in pectolinarigenin-caused inhibition of STAT3 signaling and biological functions.

### Pectolinarigenin inhibits osteosarcoma cells proliferation, colony formation and induces apoptosis in osteosarcoma cell lines

The activated STAT3 pathway has key roles in cell growth, survival and apoptosis in human cancers.^6^ To evaluate the anti-proliferative effect of pectolinarigenin, we performed MTS cell proliferation assay using a panel of osteosarcoma cells. Pectolinarigenin effectively decreased the viability of 143B, MG63.2, HOS and MG63 cells in a concentration-dependent manner (Figure 3a). Colony formation is considered to be well simulated, the pathological process of tumor development *in vivo*. We analyzed clonogenicity of various osteosarcoma cell lines after treatment with pectolinarigenin. As shown in Figure 3b, pectolinarigenin treatment resulted in a marked decrease in colony numbers. In addition, we examined the pro-apoptotic propensity of pectolinarigenin. Flow cytometry analysis showed that a large percentage of 143B cells underwent apoptosis after pectolinarigenin exposure (Figure 3c). We then investigated the effect of pectolinarigenin on STAT3 downstream target genes, which are closely related to tumor cell growth, survival and apoptosis. An immunoblotting assay revealed the protein level of STAT3 downstream targets cyclin D1, Survivin, B-cell lymphoma 2 (Bcl-2), B-cell lymphoma extra-large (Bcl-XL) and myeloid cell leukemia 1 (Mcl-1) was significantly reduced by pectolinarigenin (Figure 3d). Collectively, these results showed pectolinarigenin inhibits osteosarcoma cells cell growth, survival and induces apoptosis via suppressing STAT3 signaling.

### Pectolinarigenin inhibits adhesion, migration, invasion and reversed EMT phenotype in osteosarcoma cells

Tumor metastasis requires precisely orchestrated regulation of multiple cellular processes that involve cell adhesion, migration and invasion. To determine whether pectolinarigenin inhibits osteosarcoma cells adhesion, migration and invasion, we used 143B and MG63.2 cells with highly invasive property to perform experiments. As shown in Figure 4a (left panel), pectolinarigenin effectively impaired osteosarcoma cell adhesion to the matrix in a dose-dependent manner. In addition, osteosarcoma cell migration and invasion were markedly blocked by pectolinarigenin (Figures 4a and b). To mimic the three-dimensional (3D) conditions similar to those observed *in vivo* during tumor cell invasion, we developed a 3D culture model. In control group, osteosarcoma cells formed 3D clusters with cells protruding into the surrounding matrix, whereas treatment with pectolinarigenin resulted in the opposite phenotypes (Figure 4c). Epithelial–mesenchymal transition (EMT) is considered to be a critical mechanism regulating the initial steps in metastatic progression.^28^ Previous studies reported STAT3 may directly mediate EMT in cancer progression.^29^ To investigate the effect of pectolinarigenin on osteosarcoma EMT, we examined EMT-associated markers. We found pectolinarigenin could significantly downregulate the expression of mesenchymal markers (N-cadherin, fibronectin and zinc-finger E-box binding homeobox 1 (ZEB1)) and upregulate epithelial cell marker E-cadherin (Figure 4d). In line with this result, an immunofluorescence (IF) assay indicated exposure to pectolinarigenin resulted in a reverse of EMT, as indicated by the decreased membrane-located N-cadherin and increased E-cadherin (Figure 4e). These results suggested that pectolinarigenin showed metastasis inhibitory effects *in vitro*, further supporting the testing of *in vivo* antimetastasis efficacy of pectolinarigenin in osteosarcoma.

### Pectolinarigenin inhibits tumor growth, metastasis and prolongs the survival of mice in a spontaneous animal model

To assess whether the biologic effect of pectolinarigenin on osteosarcoma is potentially clinically relevant, we detected the *in vivo* efficacy of pectolinarigenin in tumor growth and metastasis in orthotopic osteosarcoma implanted mice. Discernable differences in tumor growth among pectolinarigenin-treated and control tumors were observed, as tumor weight was markedly relived in pectolinarigenin treatment groups compared with control group (Figure 5a). We also found the lung weight of control mice was drastically increased because of metastasis burden (Figure 5b). In high-dose group, metastasis nodules were hardly observed in lungs (Figure 5c, left panel). The number of lung metastasis was significantly reduced in mice that received pectolinarigenin (Figure 5c, right panel). Approximately 90% of mortality from cancer patients is attributable to metastases. To detect whether the metastasis suppression effect of pectolinarigenin could yield a survival benefit, the survival rate was calculated. Our data showed pectolinarigenin remarkably improved overall survival of tumor bearing mice. On day 32, all the mice had died in control group, whereas only one mouse died in high-dose pectolinarigenin treatment group (Figure 5d). Moreover, in agreement with our *in vitro* results, xenografts treated with pectolinarigenin displayed a lower level of STAT3 p-Tyr705 in comparison with control group (Figures 5e and f). We also found pectolinarigenin induced SHP-1 expression and downregulated STAT3 downstream genes (Survivin, Bcl-2 and Bcl-XL) expression (Figure 5f). Altogether, these *in vivo* results showed that pectolinarigenin suppresses osteosarcoma growth and metastasis by blocking STAT3 signaling.

### Pectolinarigenin inhibits tumor growth in a patient-derived osteosarcoma xenograft animal model

Patient-derived xenograft (PDX) models may be superior to traditional cell line xenograft models of cancer because they maintain more similarities to the parental tumors.^30^ We subcutaneously transplanted the second generation of patient-derived osteosarcoma in nude mice. We detected significant difference in tumor growth among pectolinarigenin-treated and control group. Grafts treated with pectolinarigenin had an average volume of 480.44 mm^3^ (20 mg/kg/2 days) and 182.84 mm^3^ (50 mg/kg/2 days) (Figure 6a). However, the average volume in control group was 776.58 mm^3^. In line with this, tumor weight was significantly reduced after pectolinarigenin administration in comparison with solvent control (Figure 6b). Immunohistochemistry assay and immunoblotting analysis of tumor tissue indicated STAT3 p-Tyr705 level decreased in pectolinarigenin treatment group compared with control group (Figures 6c and d). Furthermore, we found pectolinarigenin induced SHP-1 expression and downregulated STAT3 downstream genes (Survivin, Bcl-2 and Bcl-XL) expression (Figure 6d). These data implied that the growth inhibitory effect of pectolinarigenin correlated with suppression of STAT3 signaling in patient-derived tumors. Altogether, these result solidly showed that pectolinarigenin possesses antitumor activity in osteosarcoma.

### The potential toxicity of pectolinarigenin on mice

To investigate the systemic potential toxicity of pectolinarigenin, male BALB/c mice received intraperitoneal (i.p.) injection of pectolinarigenin (50 mg/kg/2 days) for 28 days. Body weight was detected once a week. Mice were killed on day 29, and the major organs were weighed and paraffin embedded for hematoxylin and eosin (H&E) staining. No significant changes in mice body and organ weight were observed after treatment with pectolinarigenin (Figures 7a and b). H&E staining revealed that pectolinarigenin showed no obvious damage to major organs including heart, lung, liver, spleen and kidney (Figure 7c). It implied that pectolinarigenin shows few side effects on the mouse body at our therapeutic concentration.

## Discussion

Constitutive activation of STAT3 has been detected in a wide range of tumor types and pharmacological inhibition of STAT3 has shown its vast potential as anticancer therapies *in vitro* and *in vivo*. In our current study, we showed that pectolinarigenin is a potent STAT3 inhibitor that inhibits osteosarcoma growth and metastasis. We found that pectolinarigenin disturbed the DNMT1/HDAC1/STAT3 complex formation in SHP-1 promoter site, thus releasing the transcription repression of SHP-1. Our results indicated the antitumor action of pectolinarigenin mainly depended on SHP-1-mediated STAT3 signaling suppression. In addition, we used cell line and patient-derived osteosarcoma animal models to reveal pectolinarigenin inhibited tumor growth and metastasis with no obvious side effects *in vivo*. Our findings provide solid evidence for the anti-osteosarcoma action and new mechanistic insight of pectolinarigenin that may aid its application in osteosarcoma intervention.

Our findings clearly displayed that pectolinarigenin inhibited STAT3 signaling. Previous studies reported inhibition of STAT3 signaling by RNA interference (RNAi), peptides, and small molecular inhibitors lead to successful suppression of tumor cell growth and metastasis.^31^ In addition, series of downstream target genes of STAT3 signaling have been identified, including that encode anti-apoptotic and proliferation-associated proteins (such as Bcl-xL, Bcl-2, cyclin D1 and Survivin).^32^ These small molecules inhibit STAT3-mediated gene regulation, block tumor cell proliferation and selectively induce apoptosis of tumor cells with activated STAT3. In this study, pectolinarigenin suppressed osteosarcoma cell proliferation and induced apoptosis, meanwhile, we also investigated pectolinarigenin downregulated STAT3 downstream proteins, such as, Bcl-xL, Bcl-2, cyclin D1 and Survivin. These founds supported that pectolinarigenin has a function on anticancer mainly because of its STAT3 signaling inhibitory activity.

Our results showed pectolinarigenin induced SHP-1 expression via promoting its transcriptional activity. SHP-1 is a tyrosine phosphatase being proposed as a candidate tumor-suppressor gene in various cancers. And it functions as an antagonist to the tumor growth and metastasis-related tyrosine kinases.^33, 34^ SHP-1 binds to JAK2 and regulates the activity of JAK2 and STAT3. It is deemed as a negative regulator of JAK2/STAT3 signaling pathway.^35^ In our results, silencing SHP-1 can rescue the reduced expression of p-STAT3 by pectolinarigenin (Figure 2f). Previous study indicated STAT3, DNMT1 and histone deacetylase 1 from transcriptional repressive complex, which could silence the expression of SHP-1.^27^ We speculate that the accumulation of SHP-1 by pectolinarigenin may be partially due to the disruption of this complex. As expected, pectolinarigenin disturbed this complex formation in SHP-1 prompter site. STAT3 is often considered as a transcription activator. However, transcription repression by STAT3 has also been reported.^36^ Our chromatin immunoprecipitation (ChIP) analysis showed STAT3 diminished in the SHP-1 promoter region after pectolinarigenin treatment. These data may imply STAT3 is a transcription repressor when binding to the promoter of the tumor suppressor. SHP-1 promoter hypermethylation would also lead to its downregulation with consequent activated phosphorylation of STAT3.^37^ We speculate the combined STAT3 and DNMT inhibition is a reasonable treatment strategy in STAT3-activated cancers.

During the process of EMT, carcinoma cells lose their epithelial characteristics, including polarity and cell–cell adhesion, and acquire a mesenchymal cell phenotype to gain invasion capacity.^38^ EMT is a critical step in order for epithelial-derived malignancies to metastasize; however, it also has vital roles for mesenchymal-derived tumor metastasis, such as osteosarcoma.^39, 40^ The reason of highly metastatic propensity of osteosarcoma may be partly due to its mesenchymal origin and osteosarcoma could be considered as a tumor that has undergone EMT. STAT3 signaling pathway has been validated to involve in tumor EMT. STAT3 promotes ZEB1 expression and downregulates E-cadherin and therefore directly mediates EMT progression in colorectal carcinoma.^41^ Indeed, we found a high level of EMT driver proteins, including N-cadherin, fibronectin and ZEB1 in osteosarcoma cell lines. However, we hardly detected E-cadherin (epithelial markers) expression in highly metastatic osteosarcoma cells at a relevant high concentration of protein (about 120 *μ*g). Our result showed pectolinarigenin significantly induced the expresson of E-cadherin in osteosarcoma cells. Reversing osteosarcoma cell EMT behavior may partly explain the reduced tumor invasion and metastasis by pectolinarigenin. These results support that pectolinarigenin serves as a novel STAT3 inhibitor that antagonizes EMT and thereby prevents osteosarcoma metastasis.

An important finding in this study is that pectolinarigenin displayed satisfactory therapeutic efficacy in animal models. Approximately 40–50% of osteosarcoma patients will develop pulmonary metastasis, and the 5-year survival rate of patients with metastases is even lower than 30%.^42^ In our orthotopic implantation xenograft animal model, we found the metastasis of tumor cells to the lungs was significantly inhibited and the survival of the mice was improved. Recent studies have suggested that the phenotype of cultured cell lines has diverged substantially from the clinical patient tumors from which they derived.^30^ Cell lines may lose their heterogeneity under the laboratory culture conditions.^43^ However, PDXs are based on the transfer of tumors directly from the patient into an immunodeficient mouse, and are of high value in the translation of cancer therapeutics into clinical settings.^30, 43^ Patient-derived human osteosarcoma xenograft animal model was applied to detect the effect of pectolinarigenin in our research. Remarkably, mice treated with pectolinarigenin showed a robust inhibition of tumor growth during the course of the experiment, compared with the control mice. We also found pectolinarigenin suppressed the expression of p-STAT3^Tyr705^ in tumor tissue, therefore mirroring our *in vitro* data. These results showed that pectolinarigenin may provide significant clinical benefits in the treatment of osteosarcoma.

Our studies suggest that pectolinarigenin possesses the inhibitory potential for osteosarcoma growth and metastasis by SHP-1-mediated STAT3 signaling inhibition. However, it remains plausible that pectolinarigenin may exhibit its anti-osteosarcoma activity through impairing/activating other signaling. Further investigations are needed to comprehensively explore the molecular mechanism of pectolinarigenin, which will help us better understand the function of pectolinarigenin on osteosarcoma. In addition, STAT3 inhibitors also have beneficial clinical therapeutic effects on several types of cancer (breast, ovarian, prostate, pancreatic, etc.), and it will be essential to determine the efficacy of pectolinarigenin against other cancer types.

## Materials and Methods

### Materials

Purified pectolinarigenin (MF: C_17_H_14_O_6_, MW: 314.28, purity > 98 %) was purchased from Shanghai Yuan Ye Biotechnology Co. Ltd (Shanghai, China). All the cell culture reagents were purchased from Invitrogen Life Technologies (Carlsbad, CA, USA). Dimethyl sulfoxide (DMSO) was obtained from Sigma-Aldrich (St. Louis, MO, USA). Matrigel was purchased from BD Bioscience (Pasadena, CA, USA). Antibodies against p-STAT3 (Y705), STAT3, histone H3, HDAC1, PTEN, N-cadherin, Zeb1, E-cadherin cyclin D1, Survivin, Bcl-2, Bcl-xl and Mcl-1 were purchased from Cell Signaling Technology Inc. (Danvers, MA, USA). Anti-DNMT1 antibody was purchased from Santa Cruz Biotechnology (Santa Cruz, CA, USA). Antibodies of SHP-1, fibronectin and SHP-2 were purchased from Abcam (Hong Kong, China). Antibody against actin was purchased from Sigma-Aldrich (Sigma-Aldrich, Inc., Shanghai, China).

### Cell lines

143B, HOS and MG63 were purchased from ATCC (Manassas, VA, USA). MG63.2 cell line was established by serially passaging the parental MG63 cells.^44^ All cells were maintained in DMEM supplemented with 10% FBS and 1% penicillin/streptomycin. Cells were maintained at 37 °C under a humidified 5% CO_2_ incubator.

### STAT3 luciferase reporter assay

The STAT3 luciferase reporter plasmid (pGMSTAT3-Luc) was used to detect STAT3 activation and obtained from Shanghai Yi Sheng Biotechnology Co. Ltd. (Shanghai, China) and procedure were carried out as previously described.^45^ 143B cells were seeded in 24-well plates 24 h before transfection. The cells were co-transfected with pGMSTAT3-Luc and pRL-SV40 (a plasmid encoding Renilla luciferase) using Lipofectamine 2000 (Invitrogen, Carlsbad, CA, USA). After 24 h, cells were treated with the indicated concentrations of pectolinarigenin for 24 h. Luciferase activity was assessed by the dual-luciferase reporter assay system (Promega, Madison, WI, USA) using a luminometer (Thermo Scientific, Waltham, MA, USA). The inhibition of STAT3 activation by pectolinarigenin was calculated as the ratio between the value of firefly and Renilla luciferase activity. Three independent experiments were carried out in triplicate.

### Western blotting

Cells and tumor tissue were lysed with radioimmunoprecipitation (RIPA) buffer (50 mmol/l Tris–HCl (pH 7.4), 150 mmol/l NaCl, 5 mmol/l EDTA, 1% Triton X-100, 1% sodium deoxycholic acid and 0.1% SDS) plus with 2 mmol/l phenylmethylsulfonyl fluoride (PMSF), 50 mmol/l NaF, 1 mmol/l Na_3_VO_4_, and protease or phosphatase inhibitor cocktail (Sigma-Aldrich, Inc.). Soluble protein lysate concentrations were determined by the BCA protein assay kit (Pierce, Rockford, IL, USA). Equal amounts of total or nuclear protein (20–120 *μ*g) were resolved on 8–12% SDS-PAGE and transferred onto polyvinylidene difluoride nitrocellulose membranes (Millipore, Billerica, MA, USA). Membranes were incubated in 5 % (w/v) bovine serum albumin (BSA/TBST) and incubated overnight at 4 °C on a shaker with specific primary antibodies. Membranes were washed with TBST and then incubated with secondary antibody (Sigma-Aldrich, Inc.) for 1 h at room temperature. After washing three times, the signal bands were visualized via chemiluminescence western blot detection reagent (ECL kit) and auto-radiographic film.

### Immunofluorescence assay

Cells grown on coverslips were exposed to different concentrations of pectolinarigenin for 24 h (for detecting STAT3 cytoplasmic-to-nuclear translocation) or 72 h (for detecting EMT-related proteins expression), fixed with 4% paraformaldehyde and permeabilized with 0.1% Triton X-100 in PBS. Samples were blocked with 1% BSA for 30 min followed by incubation with indicated primary antibodies at 4 °C overnight. After washing three times, cells were probed with Alexa Fluor 488 secondary antibody for 1 h at room temperature. The nuclei were stained by 4′, 6-diamidino-2-phenylindole (DAPI). Images were acquired with a confocal microscope (Leica, Wetzlar, Germany).

### Electrophoretic mobility shift assay

EMSA was performed using Odyssey Infrared STAT3 EMSA Kit (LI-COR Biosciences, Lincoln, NE, USA) following the manufacturer's protocol. In brief, 143B cells were pretreated with pectolinarigenin and stimulated with IL-6. Nuclear extracts were prepared and incubated with STAT3 IRDye 700 infrared dye-labeled oligonucleotides: 5′-GATCC**TTCTGGGAATT**CCTAGATC-3′ and 3′-CTAGG**AAGACCCTTAA**GGATCTAG-5′ (boldface indicates STAT3-binding sites) in reaction buffers, for 30 min at 37 °C. The protein–DNA complex was applied to native polyacrylamide gels. The gels were visualized with Odyssey infrared system.

### RT-PCR

RNA samples from cells were prepared using Trizol (Invitrogen, Carlsbad, CA, USA) according to the manufacturer's protocols. Total RNA (1 *μ*g) was converted to cDNA using oligo dT primer. The relative expression of SHP-1 was analyzed by RT-PCR with actin as an internal control. The primer sequences used for SHP-1 were 5′-GAGAACGCTAAGACCTACATCG-3′ and 5′-CAGTATGGGACG CATTTGTT-3′. PCR products were separated on 1.5% agarose gel and then stained with GelRed. Three independent experiments were carried out in triplicate.

### Co-immunoprecipitation

Co-immunoprecipitation was performed as previously reported.^46^ 143B cells were treated with or without pectolinarigenin for 24 h as indicated concertrations. Equal amount of proteins was incubated with anti-STAT3 or anti-DNMT1 antibodies overnight at 4 °C. The immunoprecipitated pellets were then incubated with protein A/G agarose beads followed by five washes with wash buffer. The eluted proteins were resolved on 8% SDS-PAGE. Three independent experiments were carried out in triplicate.

### ChIP assay

ChIP assay was performed as previously described.^46^ 143B cells were cross-linked in 1% formaldehyde in PBS for 10 min, followed by adding glycine to quench unreacted formaldehyde. Cell lysates were then collected with cold lysis buffer for ChIP and sonicated to obtain chromatin with an average fragment size of 500 bp. The chromatin samples were precleared with protein A/G agarose/salmon sperm DNA beads for 1 h and then immunoprecipitated with indicated antibodies. The immuoprecipitates were then incubated with protein A/G agarose beads for 2 h. After five sequential washes, the protein–DNA complex was eluted with elution buffer plus proteinase K and the cross-links were reversed at 65 °C for 12 h. DNA was extracted with phenol–chloroform. Immunoprecipitated DNA was analyzed by real-time PCR, and PCR products were separated on 1.5% agarose gel and stained with GelRed. The sequences of the primers used in the ChIP assay were as follows: 5′-AGGGTTACTTCCTGGTCTGTTC-3′ and 5′-ACGTCGGAGTGAGCATCAAC-3′.

### MTS cell viability assay

MTS cell viability assay was performed according to the manufacturer's instructions (Promega). In brief, osteosarcoma cells (5 × 10^3^ per well) were seeded into 96-well plates 24 h before pectolinarigenin treatment. Forty-eight hours after pectolinarigenin exposure, Aqueous One solution were added and the absorption was acquired at 490 nm by a microplate spectrophotometer (Thermo Scientific). Three independent experiments were carried out in triplicate.

### Wound-healing migration assay

Wound-healing migration assay was performed as previously described.^47^ Osteosarcoma cells were seeded into six-well plates and when growing into full confluence, a ‘wound' was created by a sterile 100 *μ*l pipette tip. Fresh medium containing different concentrations of pectolinarigenin was subsequently added. After 12 h, cells were fixed with 4% paraformaldehyde, and images were obtained by an inverted microscope (Olympus, Tokyo, Japan). Migrated cells were counted manually. Three independent experiments were carried out in triplicate.

### Transwell invasion assay

Transwell invasion assay was conducted using a modified Boyden chamber coated with Matrigel as previously described.^48^ Osteosarcoma cells were resuspended at 5 × 10^4^ cells in 100 *μ*l medium with or without indicated concentrations of pectolinarigenin and added to each transwell insert. In all, 500 *μ*l of growth medium was placed in each bottom well. Ten hours after seeding, invaded cells in the lower side of the insert were fixed with 4% paraformaldehyde and stained with 0.1% crystal violet. Images were acquired by an inverted microscope (Olympus) and invaded cells were counted manually. Three independent experiments were carried out in triplicate.

### Three-dimensional on-top assay

Three-dimensional on-top assay was conducted as previously described.^46^ Briefly, 80 *μ*l Matrigel solution per well was added into a 48-well plate and left in 37 °C for 30 min to solidify. In all, 1.5 × 10^4^ 143B cells were resuspened in 100 *μ*l DMEM and seeded on solidified Matrigel. After 15 min, 100 *μ*l DMEM containing 10% Matrigel as well as indicated concentrations of pectolinarigenin was added on top of the plated culture. The on-top Matrigel-medium mixture was replaced every 2 days. Three independent experiments were carried out in triplicate.

### siRNA-mediated knockdown

143B cells were seeded in a six-well plate 24 h before transfection. siRNA duplex targeting SHP-1 were transfected using Lipofectamine 2000 (Invitrogen Life Technologies) according to the manufacturer's protocols. The sequences targeting SHP-1 were as follows: 5′-GCAGGAGGUGAAGAACUUG-3′ (siRNA-1) and 5′-CCAGUUCAUUGAAACCAUTAA-3′ (siRNA -2).

### Establishment of SHP-1 overexpression cell line

Human SHP-1 was cloned into vector pcDNA3.1 to generated SHP-1 expression plasmid. 143B cells were transiently transfected with the pcDNA3.1-SHP-1 plasmid using Lipofectamine 2000 according to the manufacturer's instruction (Invitrogen, Gaithersburg, MD, USA). To produce stably transfected cells, cells were selected in the presence of G418 (1.0 mg/ml).

### Mice xenograft models

All animal care and experimental studies were conducted according to the guidelines and approval of the Animal Investigation Committee of the Shanghai First People's Hospital, Shanghai Jiao Tong University School of Medicine. Male BALB/c athymic nude mice and BALB/c mice were bred and maintained at the animal center in Shanghai First People's Hospital (21 °C, 55% humidity, on a 12-h light–dark cycle).

For the spontaneous growth and metastasis model, 143B tumor cells (1 × 10^6^) were suspended in sterile 20 *μ*l PBS and implanted into the medullary cavity of tibia of each mouse. One week after cell inoculation, the mice were randomly divided into three groups (*n*=6 per group) and received i.p. injection of pectolinarigenin (20 mg/kg/2 days and 50 mg/kg/2 days) as compared with mice injected with DMSO (control group). After 24 days, all mice were killed. The posterior limb with tumors and lungs were finely excised for further study. Tumor weight was measured and lung metastasis nodules numbers were counted using a dissecting microscope by three individuals who do not have personal biases with the current experiment. Tumor tissues were snap frozen in liquid nitrogen for western blotting. Another independent animal experiment was performed to determine survival curve.

The patient-derived human osteosarcoma xenografts (PDXs) animal model was conducted according to previously described procedures.^49^ Briefly, surgical specimens from patients undergoing removal of primary osteosarcoma tumors at Shanghai First People's Hospital were implanted s.c. into nude mice. When the tumors have successfully engrafted, tumor samples were passaged into subsequent generations of nude mice for the following studies. On day 14, the mice were randomized into three groups and given i.p. injection of pectolinarigenin (20 mg/kg/2 days and 50 mg/kg/2 days) as compared with mice injected with DMSO (control group). Tumor volume was measured by a digital caliper once per week. Tumor volume was determined using the following formula: (length × width^2^) × 0.52. After treatment for 28 days, all the mice were killed. The tumors were removed and prepared for western blot.

### H&E staining

Hearts, livers and other organs were freshly collected from mice when the experiments terminated and fixed in 4% paraformaldehyde overnight before paraffin embedding. In all, 4 *μ*m sections were then deparaffinization for H&E staining and representative images were acquired with a Leica microscope.

### Statistical analysis

Data are presented as mean±S.D. A Student's *t*-test was used to compare two groups (*P*<0.05 was considered significant) unless otherwise indicated. All experiments were performed at least three times.

## Figures and Tables

**Figure 1:** Pectolinarigenin inhibits STAT3 activity in osteosarcoma. (**a**) 143B cells were transfected with STAT3 luciferase reporter gene plasmid and treated with different concentrations of pectolinarigenin for 24 h. The results were normalized to the Renilla luciferase activity (**P<0.01; ***P<0.001). (**b**) Chemical structure of pectolinarigenin. (**c**) A panel of osteosarcoma cell lines was exposed to the indicated concentrations of pectolinarigenin for 24 h. Cells were then lysed and applied to immunoblotting with the indicated antibodies. Actin was used as an internal control. (**d**) Osteosarcoma cell lines were pretreated with the indicated concentrations of pectolinarigenin for 24 h and then stimulated with IL-6 (20 ng/*μ*l) for 30 min. Whole-cell extracts were prepared and subjected to western blot using the indicated antibodies. (**e**) 143B cells were seeded on gelatin-coated coverslips and pretreated with pectolinarigenin for 24 h followed by stimulating with IL-6 (20 ng/*μ*l) for 30 min. The coverslips were examined by a confocal microscopy. Anti-STAT3 antibody (green) was used to locate endogenous STAT3. Cell nuclei were stained with 4′, 6-diamidino-2-phenylindole (DAPI). Scale bar, 20 *μ*m. (**f**) 143B cells were treated with pectolinarigenin for 24 h, and the cytoplasmic and nuclear extractions were subjected to immunoblotting to detect the level of STAT3. (**g**) 143B cells were pretreated with pectolinarigenin and stimulated with IL-6. An EMSA assay was performed to analyze STAT3 DNA-binding activity

**Figure 2:** SHP-1 has an important role in pectolinarigenin-mediated STAT3 Tyr705 phosphrylation repression. (**a**) 143B and MG63.2 cells were treated with vanadate (100 *μ*M) and pectolinarigenin (20 *μ*M). Whole-cell lysates were prepared and applied to immunoblotting with an anti-phospho-STAT3 (Y705) antibody. (**b**) 143B cells were exposed to increasing concentrations of pectolinarigenin. SHP-1, SHP-2 and PTEN were probed by a western blot assay. (**c**) 143B cells were treated with pectolinarigenin for 24 h and then analyzed for SHP-1 mRNA expression by RT-PCR. (**d**) 143B cells were treated with pectolinarigenin and nuclear extracts were prepared. The immunoprecipitation assay was performed using indicated antibodies. (**e**) 143B cells were incubated with pectolinarigenin and the proteins were cross-linked with DNA and analyzed by a quantitative ChIP assay with indicated antibodies. (**f**) 143B cells were transfected with SHP-1 siRNA and treated with pectolinarigenin (20 *μ*M). Western blot analysis was used for detecting phospho-Tyr705-STAT3 expression. Cell viability was measured by a MTS assay (**P<0.01). (**g**) SHP-1 was overexpressed in 143B cells. Cells were then incubated with 20 *μ*M pectolinarigenin. Phospho-Tyr705-STAT3, STAT3 and SHP-1 were detected by a western blot assay. Cell viability was measured by a MTS assay (***P<0.001)

**Figure 3:** Pectolinarigenin inhibits osteosarcoma cells proliferation, colony formation, and induces apoptosis in osteosarcoma cell lines. (**a**) Osteosarcoma cells (143B, MG63.2, HOS and MG63) were treated with increasing concentrations of pectolinarigenin for 48 h and a MTS assay was performed (**P<0.01; ***P<0.001). (**b**) Osteosarcoma cells were seeded into six-well plates and treated with or without 10 *μ*M pectolinarigenin for a week. Colonies were then fixed and stained with 0.1% crystal violet. Images were taken by an invert microscope (Leica). Colony numbers were counted manually (*P<0.05; **P<0.01; ***P<0.001). (**c**) 143B cells were treated with pectolinarigenin at the indicated doses for 48 h. Apoptotic cells were labeled with Annexin V and PI and analyzed by flow cytometry (*P<0.05; **P<0.01). (**d**) A western blot assay was used to detect the protein level of STAT3 target genes after pectolinarigenin exposure

**Figure 4:** Pectolinarigenin inhibits adhesion, migration, invasion and reversed EMT phenotype in osteosarcoma cells. (**a**) Left panel, adhesion assay. 143B and MG63.2 cells were pretreated with various concentrations of pectolinarigenin for 12 h. Cells were trypsinized, and seeded on a fibronectin coated 96-well plate. After 15 min, non-adherent cells were removed and adherent cells were stained with 0.1% crystal violet. The precipitates were dissolved in 30% acetic acid, and the absorption at 590 nm was acquired. Middle panel, wound-healing migration assay. 143B and MG63.2 cells were seeded into six-well plates and left to grow to full confluence. Cells were scratched to create a wound and exposed to different concentrations of pectolinarigenin. Images were acquired after 12 h. Cell migration was quantified manually. Right panel, invasion assay. 143B and MG63.2 cells were resuspended in serum-free medium and seeded into the upper chamber of the transwell inserts precoated with Matrigel. Complete medium containing different concentrations of pectolinarigenin were added in the bottom well. After 12- h incubation, images were obtained. Cell invasion was quantified manually. (**b**) Representative images of migration (left panel) and invasion assay (right panel). Scale bar, 100 *μ*m. (**c**) 3D culture assay. 143B cells were seeded onto solidified Matrigel. Complete medium containing 10% Matrigel and increasing concentrations of pectolinarigenin were added on top of the cells. Four days later, cells were photographed using an inverted microscope. Scale bar, 100 *μ*m. (**d**) 143B and MG63.2 cells were incubated with increasing doses of pectolinarigenin for 72 h. EMT-related markers were probed by a western blot assay. (**e**) 143B cells were treated with pectolinarigenin at the indicated doses. Cells were examined for the expression of N-cadherin (green) and E-cadherin (green) by immunofluorescence staining. Nuclei were stained with DAPI (blue). Scale bar, 10 *μ*m

**Figure 5:** Pectolinarigenin inhibits tumor growth, metastasis and prolongs survival in an orthotopic osteosarcoma mouse model. (**a**) 143B cells were injected into the medullary cavity of tibia of the tested mice. Twenty-four days after pectolinarigenin administration, mice in different groups were killed and the posterior limb with tumors was weighed (*P<0.05; ***P<0.001). (**b**) Lungs in different groups were excised and weighed (*P<0.05; ***P<0.001). (**c**) Lung colonization was visualized by a dissecting microscope and lung metastasis nodules were counted manually (***P<0.001). In all, 4 *μ*m sections of lungs were subject to H&E staining (left lower panel). Scale bar, 100 *μ*m. (**d**) Overall survival rate in the orthotopic osteosarcoma mouse model. (**e**) Primary tumors were removed, fixed and paraffin embedded at the end of the experiment. Four micrometer (4 *μ*m) sections were analyzed by IHC using an anti-phospho-STAT3 (Y705) antibody. Scale bar, 100 *μ*m. (**f**) Primary tumors were lysed and subjected to immunoblotting with indicated antibodies. Actin was used as a loading control

**Figure 6:** Pectolinarigenin inhibits tumor growth in a patient-derived osteosarcoma xenograft (PDX) animal model. (**a**) Representative images of patient-derived osteosarcoma grafts removed from mice after administration of pectolinarigenin for 28 days (left panel). Summary results of the PDX tumor volume in control group and pectolinarigenin-treated group (***P<0.001) (right panel). (**b**) PDX tumor weight in each group was measured (***P<0.001). (**c**) Patient-derived grafts were fixed and paraffin embedded. Four micrometer (4 *μ*m) sections were analyzed by IHC using an anti-phospho-STAT3 (Y705) antibody. Scale bar, 100 *μ*m. (**d**) PDX tumor was lysed and applied to immunoblotting with with indicated antibodies. Actin was used as a loading control

**Figure 7:** The potential toxicity of pectolinarigenin on mice. (**a**) Pectolinarigenin was administrated at the dose of 50 mg/kg/2 days for 28 days. Mice body weight was monitored once a week. (**b**) Major organs weight was evaluated when the experiment terminated. NS, no significance. (**c**) Major organs from control group and pectolinarigenin-treated group were stained with H&E. Scale bar, 100 *μ*m

## Abbreviations

STAT3: signal transducer and activator of transcription 3
JAK2: Janus kinase 2
BCL-2: B-cell lymphoma 2
BCL-XL: B-cell lymphoma extra-large
Mcl-1: myeloid cell leukemia 1
i.p.: intraperitoneal injection
VEGF: vascular endothelial growth factor
XIAP: X linked inhibitor of apoptosis protein
MMPs: matrix metalloproteinases
IL-6: interleukin-6
PTEN: phosphatase and tensin homolog
DNMT1: DNA methyltransferase 1
HDAC1: HDAC1 histone deacetylase 1
siRNA: small interfering RNA
ChIP: chromatin immunoprecipitation
EMSA: electrophoretic mobility shift assay
EMT: epithelial–mesenchymal transition
ZEB1: zinc-finger E-box binding homeobox 1
H&E: hematoxylin–eosin
